The article "An Extensive Set of Kinematic and Kinetic Data for Individuals with Intact Limbs and Transfemoral Prosthesis Users" was published in 2020. Journal: Appl Bionics Biomech.

# An Extensive Set of Kinematic and Kinetic Data for Individuals with Intact Limbs and Transfemoral Prosthesis Users

**DOI:** 10.1155/2020/8864854

**Published:** 2020-11-09

**Authors:** Seyed Fakoorian, Arash Roshanineshat, Poya Khalaf, Vahid Azimi, Dan Simon, Elizabeth Hardin

**Affiliations:** ^1^Department of Electrical Engineering and Computer Science, Cleveland State University, Cleveland, Ohio 44115, USA; ^2^Department of Electrical Engineering and Computer Engineering, University of Arizona, Tucson, AZ 87721, USA; ^3^Department of Mechanical Engineering, Cleveland State University, Cleveland, Ohio 44115, USA; ^4^Department of Electrical Engineering and Computer Engineering, Georgia Institute of Technology, Atlanta, GA 30313, USA; ^5^Motion Study Laboratory, Cleveland VA Medical Center, Cleveland, Ohio 44106, USA

## Abstract

This paper introduces an extensive human motion data set for typical activities of daily living. These data are crucial for the design and control of prosthetic devices for transfemoral prosthesis users. This data set was collected from seven individuals, including five individuals with intact limbs and two transfemoral prosthesis users. These data include the following types of movements: (1) walking at three different speeds; (2) walking up and down a 5-degree ramp; (3) stepping up and down; (4) sitting down and standing up. We provide full-body marker trajectories and ground reaction forces (GRFs) as well as joint angles, joint velocities, joint torques, and joint powers. This data set is publicly available at the website referenced in this paper. Data from flexion and extension of the hip, knee, and ankle are presented in this paper. However, the data accompanying this paper (available on the internet) include 46 distinct measurements and can be useful for validating or generating mathematical models to simulate the gait of both transfemoral prosthesis users and individuals with intact legs.

## 1. Introduction

A variety of kinematic and kinetic data can be collected during human motion with a well-equipped gait lab. A rich and well-organized human motion data set can enable research in biomechanics and bio-inspired control systems and signal processing. To develop bio-inspired control systems, mimicking the reactions and motions of a subject with intact legs is critical. For example, such data can be used for the design of human-like prosthesis control Moore et al. [1]. These data can also be used to verify controllers that have been designed by other means, such as those constructed from first principles Geyer and Herr [2]. Furthermore, from a medical perspective, gait data analysis can be used to identify the overactive or underactive muscles, potential injuries, and walking inefficiency Keenan et al. [3]; Avni [4].

The article "An Extensive Set of Kinematic and Kinetic Data for Individuals with Intact Limbs and Transfemoral Prosthesis Users" was published in 2020. Journal: Appl Bionics Biomech.

Human gait data from thousands of human subjects already exist, but the majority of these data are not publicly available. There are some notable gait data sets and databases that are publicly available. In 1990, David Winter published a normative gait data set that is widely used in biomechanical studies Winter [5]. These data include only a few subjects and only a small number of gait cycles per subject, but this small gait data set has been important for developing design specifications, such as in powered prosthetic control Sup et al. [6]. The International Society of Biomechanics has maintained a website International Society of Biomechanics [7] since 1995 that includes data sets that are available for download. Another website, the CGA normative gait database Kirtley [8], curates and shares normative clinical gait data from multiple labs, which have been used in several research studies. The repeatability of kinematic, kinetic, and electromyographic data was investigated in Kadaba et al. [9], where 40 adult subjects with intact limbs were evaluated three times on each of three different test days while walking at their preferred speed. That research was followed by the development of a simple external marker system and algorithms for computing lower extremity joint angle motion during level walking (VICON) Kadaba et al. [10]. The effect of walking speed on gait was considered in Schwartz et al. [11], where three-dimensional gait data was collected on 83 children (ages 4-17 years) who were given general instructions to walk at several speeds during a single test session: very slow, slow, self-selected comfortable (free), and fast. Children's gait was also studied in Bovi et al. [12], which includes data from both children and adults (ages 6-72 years) in different gait modes, such as normal walking, toe walking, heel walking, step ascent, and step descent.

More recent examples of biomechanists sharing their data through publication include the University of Wisconsin at LaCrosse, which has an easily accessible normative gait data set from 25 subjects with lower extremity marker data from multiple gait cycles, and force plate measurements from a single gait cycle Willson and Kernozek [13]. Other recent research van den Bogert et al. [14]; Moore et al. [1] includes the availability of full-body joint kinematics and kinetics from multiple subjects walking on an instrumented treadmill. That research includes over 7.5 hours of gait data from 15 subjects with intact legs and includes over 25,000 gait cycles. Those data include both perturbed and unperturbed gait cycles; perturbed gait cycles included random treadmill variations to emulate pushing the subject. Other research Fukuchi et al. [15] includes a dataset of 3D walking kinematics and kinetics from young and older adults with two intact legs at a range of gait speeds in both treadmill and overground environments. The most recent research Hood et al. [16] includes 18 transfemoral prosthesis users walking at various speeds. This data set was collected using a 10-camera motion capture system and an instrumented treadmill.

The article "An Extensive Set of Kinematic and Kinetic Data for Individuals with Intact Limbs and Transfemoral Prosthesis Users" was published in 2020. Journal: Appl Bionics Biomech.

There have been many gait studies, but relatively few are publicly available at no monetary cost. Many gait data sets are not freely accessible Tirosh et al. [17], although there are notable exceptions Kirtley [8]. The lower body kinematic data of single gait cycles from over 100 subjects, which include a substantial amount of raw data, was published in Yun et al. [18] but accessing the data requires a monetary cost. In addition, a large gait database comparison, including one database with kinematic data of 409 gait cycles of children from 1 to 7 years old, is discussed in Chester et al. [19]. There are also some purely visual gait data sets, like the one in Makihara et al. [20], which contains videos of subjects walking on a treadmill. This database is tightly secured with an extensive release agreement for reuse.

All gait data that are currently available suffer from one or more limitations such as too few subjects, gait cycles, or gait types, which limit the possibility of using the data for prosthesis design or other human-machine research. Other data sets have restrictive licensing conditions. Currently available data mostly come from humans with two intact legs during normal walking on level ground. Although many transfemoral prosthesis users participated in Hood et al. [16], they only collected walking data and other routine activities were not considered. In Bergmann et al. [21], only contact forces in the hip joint were measured for four patients who had hip implants. They collected data from routine activities but the data are not publicly available.

In this paper, an extensive set of data is presented from human motion in different activities of daily living. Data were collected from five individuals with intact limbs and two transfemoral prosthesis users. The subjects walked at three different speeds on a force plate-instrumented treadmill. The key feature of the data we collected is that they are from many activities of daily living, such as level walking, walking up and down a five-degree ramp, stepping up and down a step, and sitting down and rising from a chair. Our results are publicly available at Fakoorian et al. [22]. We invite other researchers to use the MATLAB source code at the website to reproduce our signal processing results for 46 kinetic and kinematic quantities, including joint angles, joint moments, and joint powers for both left and right legs.

The article "An Extensive Set of Kinematic and Kinetic Data for Individuals with Intact Limbs and Transfemoral Prosthesis Users" was published in 2020. Journal: Appl Bionics Biomech.

## 2. Methods

Five individuals with intact limbs and two transfemoral prosthesis users participated in the study. The research site was the Motion Studies Laboratory (MSL) at the Cleveland Department of Veterans Affairs Medical Center (VAMC) in Cleveland, Ohio, whose IRB approved the study. The average of age, height, and weight of the subjects with intact limbs are 26 years, 182.1 cm, and 79.8 kg, respectively. Additional information about the subjects with intact limbs can be found in Table 1.

The prosthesis users had an average age of 48 years, an average height of 175.8 cm, and an average weight of 89.2 kg. The first prosthesis user used an X2 microprocessor knee (Ottobock, Duderstadt, Germany) with a Triton foot, and the second prosthesis user used a Plie 3 microprocessor knee (Freedom Innovations, Irvine, California) with a hydraulic foot. Both prosthesis users had their intact limb on the left side and their prosthesis on the right side.  Table 2 gives additional details about the transfemoral prosthesis users.

Joint angles and torques were computed from the construction of an individualized human body model comprising 18 body segments and 46 kinematic degrees of freedom. The human body model was based on 47 markers affixed in standard anatomical locations on each individual human subject (Motek, Amsterdam, NL). Acronym definitions of 47 markers are listed in Table 3. A lower body model shown in Figure 1 was used for some participants due to their time restrictions Moore et al. [1]; van den Bogert et al. [14]. The kinetic data meet the collection and processing guidelines from the International Society of Biomechanics Derrick et al. [23].

Data were collected under the following conditions: (1) walking at three different speeds on level ground, (2) walking up and down a ramp with a five-degree slope, (3) stepping up onto a standard-height step and stepping down from the same step, and (4) sitting down in a standard height chair and standing up from the chair. A 16-camera motion capture system (Vicon, Oxford, UK) was used to record the marker positions at 100 Hz. Ground reaction force (GRF) was sampled at 1000 Hz from several force plates (OR6-7-OP and AccuGait, AMTI, Watertown, Massachusetts; Forcelink BV, Culemborg, Netherlands). Data were collected during standing to initialize each individual human body model. Raw data were filtered with a 6 Hz low-pass filter (second order Butterworth). Finally, inverse modeling was used to calculate kinetic and kinematic data van den Bogert et al. [14]. Part of the experimental setup for both the participants with intact legs and transfemoral prosthesis user participants during the walking data collection is shown in Figure 2.

The article "An Extensive Set of Kinematic and Kinetic Data for Individuals with Intact Limbs and Transfemoral Prosthesis Users" was published in 2020. Journal: Appl Bionics Biomech.

As shown in Figure 3, one force plate was used for collecting the ramp walking data, thus one step of GRF data exists per ramp walking trial in this repository. The joint kinematics presented in this paper are for a sample of joints, and readers can download and plot additional joint kinematic as well as kinetic data Fakoorian et al. [22].

Stepping up and down trials are shown in Figure 4. Each trial consisted of stepping up on, or down from, the force plate. One force plate was embedded on the top step and captured either the left or the right foot when stepping up; two force plates were embedded in the ground and captured either the left or right foot upon stepping down.

In the sit-to-stand activity, shown in Figure 5, we collected data during the sit-to-stand transition and also during the stand-to-sit transition. We collected GRF data from two force plates, one under each foot, as shown in Figure 5.

During treadmill walking, shown in Figure 2, GRFs were collected at 1000 Hz using two force plates embedded under the belts of the treadmills (ADAL3DM-F-COP-Mz, Techmachine, France; Forcelink, Motek Medical BV, Amsterdam, NL). Research participants walked on the treadmill while data were recorded for ten, 30-second periods. Kinematic and kinetic data were collected at each subject's preferred walking speed, which was determined using previously published methods Dingwell and Marin [24], and which allowed for acclimating to the treadmill. Data were also collected at slower than preferred speed and faster than preferred speed. All of the research participants had previous treadmill experience.

## 3. Results

In this section, results are presented for the joint kinematics and kinetics of each subject. Several movement types were collected for every participant.  Table 4 presents the number of trials (repetitions) collected for ramp walking, stepping up and stepping down, and sit-to-stand and stand-to-sit.  Table 5 shows the number of trials for walking at different speeds for participants with intact limbs (AB01-AB05). Walking speed transition data were collected for the transition from standing to fast walking (1.5 m/s), and vice versa, but only for AB02 (37 trials). For the prosthesis user participants, Table 6 shows the number of trials for each walking speed and for each type of gait transition.

Hip flexion, knee flexion, and ankle plantar flexion for selected gait types and subjects are plotted, but additional data is available for all three axes of motion Fakoorian et al. [22]. These results are provided for the right leg for each subject, except we plot data for the left leg for step mode.  Figure 6 shows the angle convention for hip flexion, knee flexion, and ankle plantar flexion. Because this is an extensive data set, only a small sample of representative data is plotted. However, the MATLAB code used to generate the results of this paper is available at Fakoorian et al. [22] and the user can plot all joint angles, joint moments, and joint powers for each trial, each subject, each activity of daily living, and either right or left leg; available data are summarized in Table 7.

The article "An Extensive Set of Kinematic and Kinetic Data for Individuals with Intact Limbs and Transfemoral Prosthesis Users" was published in 2020. Journal: Appl Bionics Biomech.

For AB01, Figure 7 shows the data from the sit-to-stand and the stand-to-sit trials. As shown, the first two trials are sit-to-stand and the remaining trials are stand-to-sit. The transition from standing to fast walking (1.5 m/s) and vice versa is presented for trials 22 and 25 for AB02 in Figure 8.  Figure 9 displays joint angles when subject AB03 is walking up and down the ramp. The figure shows that there were four gait cycles because eight steps were collected during each ramp trial. The two middle gait cycles occurred while the subject walked on the ramp. For subject AB04, Figure 10 shows the average and standard deviation of the sagittal plane joint angles and torques during preferred-speed walking, and Figure 11 shows the average and standard deviation of vertical GRF.  Figure 12 shows joint angles from the stepping up and stepping down trials for subject AB05. The step-up data is from trial 4 and is shown in the left column of the figure. The step-down data is from trial 5 and is shown in the right column of the figure. In both trials, the right leg is the leading leg and the left leg is the trailing leg.

Figure 13 shows the joint angles and torques (mean and standard deviation) for the right leg (prosthesis side) of a transfemoral prosthesis user (PR01), trial 3, over a total of 30 strides. The data are from walking at their preferred speed of 0.8 m/s. Moreover, Figure 14 shows the vertical GRF (mean and standard deviation) for the same trial.  Figure 15 shows the joint angles during the transition from slow walking (0.6 m/s) to fast walking (1.1 m/s), and vice versa, for prosthesis user PRO2. These data are shown in the figure for trials 21 and 23, respectively.

Next, we compare the spatiotemporal gait parameters between the participants with intact limbs and the transfemoral prosthesis users at different walking speeds. A scatter plot combined with a box plot is used to visualize the gait parameters in Figures 16–18. Although the gait speed of each subject is different, scatter plots show the average of the gait parameters for each individual trial for each subject, while the box plots show the ranges of the parameters. The results are distinguishable based on the gait speed of each subject. The gait parameters include stride frequency, stride length, and stride width.

The article "An Extensive Set of Kinematic and Kinetic Data for Individuals with Intact Limbs and Transfemoral Prosthesis Users" was published in 2020. Journal: Appl Bionics Biomech.

## 4. Discussion

### 4.1. Sit-to-Stand and Stand-to-Sit

In Figure 7, the middle figure shows that during the sit-to-stand transitions the knee angle gradually decreases from about 90 degrees to 0 degrees, while the converse is true for the stand-to-sit transitions, as expected. The left figure shows that the hip flexion in the sitting position is about 50 degrees (trials 1 and 2); when the subject starts standing up the hip flexion first increases as the subject leans forward to provide himself with momentum to begin standing; the angle then decreases until it reaches about -10 degrees in the standing position. Conversely, for the stand-to-sit transition, the hip flexion starts at about -10 degrees in the standing position (trials 3-5); when the subject starts sitting down the hip flexion first increases until the subject achieves contact with the seat of the chair and then decreases as the subject settles into a comfortable sitting position at around 50 degrees. As expected, and as shown in the right figure, the ankle motion has a smaller range of motion than the hip during both the sit-to-stand and the stand-to-sit transition. The variation of the ankle angle is only 15±2 degrees for all trials and is generally in dorsiflexion (≤90 degrees). The ankle angle is slightly plantar flexed, ≃80 degrees in the standing position and at a neutral angle, ≃90 degrees in the sitting position.

### 4.2. Transition from Standing to Walking

In Figure 8, when the subject walked at 1.5 m/s, maximal hip flexion was 35 degrees, maximal knee flexion was 67 degrees, and maximal ankle angle was -76 degrees (14 degrees of plantar flexion). While transitioning from fast walking to standing, the step frequency gradually decreased until the joint angles reached standing values of approximately 9 degrees, 9 degrees, and -96 degrees, respectively.

### 4.3. Ramp Walking

In Figure 9, the subject's hip flexion and ankle plantar flexion were greater when the subject walked up the ramp compared to when the subject walked down the ramp. However, knee flexion while walking down the ramp appears to be about the same as knee flexion while walking up the ramp. The first and fourth gait cycles occurred during level-ground walking before and after the ramp. As expected, the peak flexion angles of the first stride during ramp-up walking were similar to the last stride during ramp-down walking, and the peak flexion angles of the first stride during ramp-down walking were similar to those of the last stride during ramp-up walking.

The article "An Extensive Set of Kinematic and Kinetic Data for Individuals with Intact Limbs and Transfemoral Prosthesis Users" was published in 2020. Journal: Appl Bionics Biomech.

### 4.4. Participants with Intact Limbs Walking at Preferred Speed

In Figure 10, the ankle torque was greater than the hip and knee torques between 20% and 60% of the gait cycle, showing the large amount of torque needed by the ankle during normal gait. Of all the joint torques, the knee torque had the largest standard deviation during the first half of the gait cycle, the stance phase, which demonstrates the relatively high stride-to-stride variation of knee torque. During most of the gait cycle and for most of the quantities shown in the figure, the standard deviations are very low, showing the high level of repeatability for this subject's gait. The knee joint has the largest range of motion and peaks at about 75 degrees 80% through the gait cycle, when the subject lifts his leg off the ground and needs more knee flexion to achieve toe clearance during the swing phase. The figure shows, as expected, that the stance phase comprises about 60% of the gait cycle.

Figure 11 shows a typical vertical GRF curve with two peaks that occur at heel strike and toe-off near the beginning and end of the stance phase. As with most of the joint angle and torque data, the GRF standard deviation is very low, showing the high level of repeatability for this subject's gait.

### 4.5. Stepping Up and Stepping Down

Figure 12 shows that when the subject stepped up, the leading leg had more hip flexion (58 degrees) and knee flexion (95 degrees) than the trailing leg (33 degrees and 78 degrees, respectively), but more ankle plantar flexion was exhibited in the trailing leg (-44 degrees vs. -74 degrees). When stepping down, the leading hip and knee joint flexion (25 degrees and 53 degrees, respectively) were smaller than during the step-up trial (58 degrees and 95 degrees, respectively), but the leading ankle joint plantar flexion during step-down (-42 degrees) was larger than during step-up (-74 degrees). When stepping down, the trailing leg knee flexion is greater than the leading leg knee flexion (95 degrees vs. 53 degrees), but the trailing leg ankle plantar flexion is less than in the leading leg (bottom right figure). As expected, knee flexion was greater than both hip flexion and ankle plantar flexion in both the leading and trailing legs during both stepping modes. Maximum knee flexion during stepping up was 95 degrees and 80 degrees for the leading and trailing legs, respectively; and during stepping down, it was 53 degrees and 96 degrees, respectively.

### 4.6. Prosthesis User Walking at Preferred Speed

In Figure 13, in agreement with previous research, there is very little knee flexion during stance Sup et al. [6]; Brandt et al. [25]. Comparing Figures 13 and 14 with Figures 10 and 11, some differences are evident between the gait of a subject with intact legs and a prosthesis user. For the prosthesis user, the standard deviations of joint angles and joint torques were greater than those of the subject with intact legs (AB04). The standard deviation of the vertical GRF is similar for both the prosthesis user and the subject with intact legs, but the average vertical GRF of the subject with intact legs is greater than that of the prosthesis user, which agrees with previous observations that prosthesis users place more weight on their intact side than on their prosthesis Koehler-McNicholas et al. [26]. That is, the maximum vertical GRF in the mid-stance phase is 930 N for the subject with intact limbs, but only 815 N for the transfemoral prosthesis user. This difference occurs in spite of the fact that AB04 and PR01 have a similar body mass (see Tables 1 and 2). The joint angle and joint torque profiles also have different ranges. Part of this difference may be due to the different walking speeds (1.1 m/s for the subject with intact legs and 0.8 m/s for the prosthesis user). Throughout the gait cycle, the hip flexion is about the same, but the knee flexion and ankle plantar flexion are smaller for PR01 than for AB04. More joint torque is also needed for all joints for AB04, especially for the knee joint after about 60% through the gait cycle.

The article "An Extensive Set of Kinematic and Kinetic Data for Individuals with Intact Limbs and Transfemoral Prosthesis Users" was published in 2020. Journal: Appl Bionics Biomech.

### 4.7. Prosthesis User Transition from Slow to Fast Walking

In Figure 15, the peak angles gradually increased during the slow-to-fast transition (left figures) and gradually decreased during the fast-to-slow transition (right figures). The knee angle had the greatest flexion of all the joints at the end of the slow-to-fast transition, when it flexed to 70 degrees (left middle figure). The ankle angle did not have much variation and its magnitude varied by less than 35 degrees peak-to-peak.

### 4.8. Comparison of Gait Parameters

One can see from Figures 16–18 that walking speed is directly related to changes in stride frequency, length, and width in the participants with intact limbs and the variations of the stride parameters change in a predictable way with walking speed. However, for the transfemoral prosthesis users, we do not see such predictable changes in the gait parameter variations with respect to walking speed. In general, the variation of the stride parameters is greater in the participants with intact limbs than in the prosthesis users, especially for stride width. The maximum stride length is about 1.8 m for the subjects with intact legs, but only 0.97 m for the prosthesis users. This could have been expected because the maximum speed of the prosthesis users is less than that of any of the subjects with intact legs.

The article "An Extensive Set of Kinematic and Kinetic Data for Individuals with Intact Limbs and Transfemoral Prosthesis Users" was published in 2020. Journal: Appl Bionics Biomech.

This paper presents an extensive human motion data set from individuals with intact limbs and transfemoral prosthesis users. These data include walking at different speeds, walking up and walking down a 5-degree ramp, stepping up and stepping down from a step, and sitting down and rising from a chair. Our data set is free and available (along with plotting software) at Fakoorian et al. [22], where the reader can reproduce the results of this paper and can also plot ground reaction forces, joint kinematics, and joint kinetics.

These data can be used for generating or validating mathematical models for the simulation of periodic human gait. They can also be useful for developing human-mimicking prosthesis controllers for prosthesis users.

## Figures and Tables

**Figure 1:** Marker placement locations on the human body. The 25 markers shown were needed for the hip, knee and ankle kinematic, and kinetic calculations, although some subjects in our study wore the full 47-marker set.

**Figure 2:** Walking kinematics and kinetics were captured on a force instrumented treadmill.

**Figure 3:** Data collection setup for the ramp walking trials.

**Figure 4:** Data collection setup for the stepping trials: the left figure shows a stepping down trial, and the right figure shows a stepping up trial by a prosthesis user participant.

**Figure 5:** Data collection setup for the sit-to-stand and stand-to-sit trials.

**Figure 6:** Angle convention for hip flexion, knee flexion, and ankle plantar flexion. The vertical axis is zero degrees and the arrows show the positive direction. In the normal standing position shown, the hip angle is 0, the knee angle is 0, and the neutral ankle angle is approximately -90 degrees.

**Figure 7:** The first two trials are sit-to-stand transitions and the other trials are stand-to-sit transitions. These results are taken from subject AB01.

**Figure 8:** The left figures show the joint angles during the transition from standing to fast walking at 1.5 m/s (trial 22), and the right figures show the transition from fast walking at 1.5 m/s to standing (trial 25). These results are taken from subject AB02.

**Figure 9:** Joint angles during walking up the ramp (trial 9) and down the ramp (trial 10). These results are taken from subject AB03.

**Figure 10:** The mean (red) and standard deviation (shaded) of joint angles and torques during preferred-speed walking. These results are from subject AB04 (Trial 3) and include 29 gait cycles.

The article "An Extensive Set of Kinematic and Kinetic Data for Individuals with Intact Limbs and Transfemoral Prosthesis Users" was published in 2020. Journal: Appl Bionics Biomech.

**Figure 11:** The mean (red) and standard deviation (shaded) of vertical ground reaction force during preferred-speed walking. These results are from subject AB04 (Trial 3) and include 29 gait cycles.

**Figure 12:** Joint angles during stepping up (left figures, trial 4) and stepping down (right figures, trial 5). The right leg is the leading leg and the left leg is the trailing leg for both trials. These results are from subject AB05.

**Figure 13:** The mean (red) and standard deviation (shaded) of joint angles and torques for transfemoral prosthesis user PRO1, trial 3, during the preferred walking speed of 0.8 m/s. The mean and standard deviation are calculated over 30 gait cycles.

**Figure 14:** The mean (red) and standard deviation (shaded) of vertical GRF for the prosthesis user PRO1, trial 3, during the preferred walking speed of 0.8 m/s. The mean and standard deviation are calculated over 30 gait cycles.

**Figure 15:** Joint angles of transfemoral prosthesis user PR02 during the transition from slow (0.6 m/s) to fast (1.1 m/s) walking (left figures), and vice versa (right figures). The left figures are taken from trial 21 and the right figures are taken from trial 23.

**Figure 16:** Stride frequency of participants with intact limbs and prosthesis users at three speeds with the normal speed being their preferred speed. The data from participants with intact limbs is shown on the left (A) and transfemoral prosthesis user data is shown on the right (T) in each pair. The figure shows the median, along with a box that bounds the first and third quartiles of the data, and whiskers that bound the entire range of the data (apart from outliers). Moreover, the scatter plot shows the average stride frequency of each trial. The data for each subject are color-coded: yellow = AB01, green = AB02, red = AB03, blue = AB04, purple = AB05, brown = PR01, and gray = PR02.

**Figure 17:** Stride length of participants with intact limbs and prosthesis users at three speeds with the normal speed being their preferred speed. The data from participants with intact limbs is shown on the left (A) and transfemoral prosthesis user data is shown on the right (T) in each pair. The figure shows the median, along with a box that bounds the first and third quartiles of the data, and whiskers that bound the entire range of the data (apart from outliers). Moreover, the scatter plot shows the average stride length of each trial. The data for each subject are color-coded: yellow = AB01, green = AB02, red = AB03, blue = AB04, purple = AB05, brown = PR01, and gray = PR02.

**Figure 18:** Stride width of participants with intact limbs and prosthesis users at three speeds with the normal speed being their preferred speed. The data from participants with intact limbs is shown on the left (A) and transfemoral prosthesis user data is shown on the right (T) in each pair. The figure shows the median, along with a box that bounds the first and third quartiles of the data, and whiskers that bound the entire range of the data (apart from outliers). Moreover, the scatter plot shows the average stride width of each trial. The data for each subject are color-coded: yellow = AB01, green = AB02, red = AB03, blue = AB04, purple = AB05, brown = PR01, and gray = PR02.

The article "An Extensive Set of Kinematic and Kinetic Data for Individuals with Intact Limbs and Transfemoral Prosthesis Users" was published in 2020. Journal: Appl Bionics Biomech.

**Table 1:** Demographic and anthropometric data for the subjects with intact limbs.

	Age	Height (cm)	Weight (kg)	Left leg length (cm)	Left knee width (cm)	Left ankle width (cm)	Right leg length (cm)	Right knee width (cm)	Right ankle width (cm)
AB01	28	180.3	80.9	90.5	9.4	6.9	90.0	9.4	6.6
AB02	23	185.4	83.2	98.0	10.8	7.6	98.0	10.4	7.5
AB03	22	185.4	80.9	86.0	9.7	7.4	85.0	9.0	7.4
AB04	37	188.0	79.9	98.5	10.4	6.8	97.5	10.4	7.0
AB05	20	171.5	73.9	89.5	9.5	7.0	89.0	9.9	6.7

**Table 2:** Demographic and anthropometric data for the subjects who were prosthesis users.

	Age	Height (cm)	Weight (kg)	Left leg length (cm)	Left knee width (cm)	Left ankle width (cm)	Right leg length (cm)	Right knee width (cm)	Right ankle width (cm)	Prosthesis type
PRO1	32	174.0	79.1	91.0	9.5	7.2	89.0	7.4	5.2	Ottobock
PRO2	64	177.6	99.2	85.5	11.4	7.6	86.0	7.4	7.4	Freedom innovations

**Table 3:** 47 marker acronym definitions Moore et al. [1].

#	Label	Name	Description
1	LHEAD	Left head	Just above the ear, in the middle.
2	THEAD	Top head	On top of the head, in line with the LHEAD and RHEAD.
3	RHEAD	Right head	Just above the ear, in the middle.
4	FHEAD	Forehead	Between line LHEAD/RHEAD and THEAD a bit right from center.
5	C7	C7	On the 7th cervical vertebrae.
6	T10	T10	On the 10th thoracic vertebrae.
7	SACR	Sacrum bone	On the sacral bone.
8	NAVE	Navel	On the navel.
9	XYPH	Xiphoid process	Xiphoid process of the sternum.
10	STRN	Sternum	On the jugular notch of the sternum.
11	BBAC	Scapula	On the inferior angle of the right scapular.
12	LSHO	Left shoulder	Left acromion.
13	LDELT	Left deltoid muscle	Apex of the deltoid muscle.
14	LLEE	Left lateral elbow	Left lateral epicondyle of the elbow.
15	LMEE	Left medial elbow	Left medial epicondyle of the elbow.
16	LFRM	Left forearm	On 2/3 on the line between the LLEE and LMW.
17	LMW	Left medial wrist	On styloid process radius, thumb side.
18	LLW	Left lateral wrist	On styloid process ulna, pinky side.
19	LFIN	Left fingers	Center of the hand. Caput metatarsal 3.
20	RSHO	Right shoulder	Right acromion.
21	RDELT	Right deltoid muscle	Apex of deltoid muscle.
22	RLEE	Right lateral elbow	Right lateral epicondyle of the elbow.
23	RMEE	Right medial elbow	Right medial epicondyle of the elbow.
24	RFRM	Right forearm	On 1/3 on the line between the RLEE and RMW.
25	RMW	Right medial wrist	On styloid process radius, thumb side.
26	RLW	Right lateral wrist	On styloid process ulna, pinky side.
27	RFIN	Right fingers	Center of the hand. Caput metatarsal 3.
28	LASIS	Pelvic bone left front	Left anterior superior iliac spine.
29	RASIS	Pelvic bone right front	Right anterior superior iliac spine.
30	LPSIS	Pelvic bone left back	Left posterior superior iliac spine.
31	RPSIS	Pelvic bone right back	Right posterior superior iliac spine.
32	LGTRO	Left greater trochanter of the femur	On the center of the left greater trochanter.
33	FLTHI	Left thigh	On 1/3 on the line between the LFTRO and LLEK.
34	LLEK	Left lateral epicondyle of the knee	On the lateral side of the joint axis.
35	LATI	Left anterior of the tibia	On 2/3 on the line between the LLEK and LLM.
36	LLM	Left lateral malleolus of the ankle	The center of the heel at the same height as the toe.
37	LHEE	Left heel	Center of the heel at the same height as the toe.
38	LTOE	Left toe	Tip of big toe.
39	LMT5	Left 5th metatarsal	Caput of the 5th metatarsal bone, on joint line midfoot/toes.
40	RGTRO	Right greater trochanter of the femur	On the center of the right greater trochanter.
41	FRTHI	Right thigh	On 2/3 on the line between the RFTRO and RLEK.
42	RLEK	Right lateral epicondyle of the knee	On the lateral side of the joint axis.
43	RATI	Right anterior of the tibia	On 1/3 on the line between the RLEK and RLM.
44	RLM	Right lateral malleolus of the ankle	The center of the heel at the same height as the toe.
45	RHEE	Right heel	Center of the heel at the same height as the toe.
46	RTOE	Right toe	Tip of big toe.
47	RMT5	Right 5th metatarsal	Caput of the 5th metatarsal bone, on joint line midfoot/toes.

The article "An Extensive Set of Kinematic and Kinetic Data for Individuals with Intact Limbs and Transfemoral Prosthesis Users" was published in 2020. Journal: Appl Bionics Biomech.

**Table 4:** The number of available trials (repetitions) is listed for each activity except walking. STS indicates stand-to-sit or sit-to-stand. See Tables 5 and 6 for the number of walking trials.

	Ramp	Step	STS
AB01	20	44	5
AB02	38	42	23
AB03	40	46	22
AB04	43	42	29
AB05	44	42	22
PRO1	33	31	21
PRO2	NA	NA	NA

**Table 5:** The number of trials (repetitions) is listed for each walking speed for the participants with intact limbs. Note that the preferred walking speed varies with each subject.

	Fast walking			Preferred speed			Slow walking		
	1.25 m/s	1.62 m/s	1.44 m/s	1 m/s	1.1 m/s	1.15 m/s	0.75 m/s	0.9 m/s	0.86 m/s
AB01	10	NA	NA	10	NA	NA	10	NA	NA
AB02	10	NA	NA	10	NA	NA	10	NA	NA
AB03	7	NA	NA	10	NA	NA	6	NA	NA
AB04	NA	7	NA	NA	6	NA	NA	6	NA
AB05	NA	NA	6	NA	NA	6	NA	NA	6

**Table 6:** The number of trials is listed for each walking speed for the prosthesis users.

	Walking speeds			Transition	Transition
	0.6 m/s	0.8 m/s	1.1 m/s	From 0.6 to 1.1 m/s	From 1.1 to 0.6 m/s
PRO1	6	3	3	NA	NA
PRO2	5	6	5	2	2

**Table 7:** This is a complete list of the kinematic and kinetic measurements that the reader can plot using the database and software at Fakoorian et al. [22]. There are a total of 46 kinematic and kinetic measurements that can be plotted for the full-body model.

Pelvis in *x* direction	Head right bend	Left/right wrist flexion
Pelvis in *y* direction	Head left twist	Left/right hand abduction
Pelvis in *z* direction	Left/right shoulder up	Left/right hip flexion
Pelvis yaw	Left/right shoulder forward	Left/right hip abduction
Pelvis forward pitch	Left/right shoulder inward	Left/right hip internal rotation
Pelvis right roll	Left/right shoulder flexion	Left/right knee flexion
Trunk flexion	Left/right shoulder abduction	Left/right ankle plantar flexion
Trunk right bend	Left/right shoulder internal rotation	Left/right foot pronation
Trunk left twist	Left/right elbow flexion	Left/right toe flexion
Head flexion	Left/right forearm pronation	

## Data Availability

Our data and the MATLAB code used to generate the results of this paper is available at http://embeddedlab.csuohio.edu/prosthetics/research/gaitdata.html
